# Pose Estimation-Assisted Dance Tracking System Based on Convolutional Neural Network

**DOI:** 10.1155/2022/2301395

**Published:** 2022-06-03

**Authors:** Jin Mu

**Affiliations:** School of Music, Jiaozuo Normal College, Jiaozuo, Henan, 454100, China

## Abstract

In the field of music-driven, computer-assisted dance movement generation, traditional music movement adaptations and statistical mapping models have the following problems: Firstly, the dance sequences generated by the model are not powerful enough to fit the music itself. Secondly, the integrity of the dance movements produced is not sufficient. Thirdly, it is necessary to improve the suppleness and rationality of long-term dance sequences. Fourthly, traditional models cannot produce new dance movements. How to create smooth and complete dance gesture sequences after music is a problem that needs to be investigated in this paper. To address these problems, we design a deep learning dance generation algorithm to extract the association between sound and movement characteristics. During the feature extraction phase, rhythmic features extracted from music and audio beat features are used as musical features, and coordinates of the main points of human bones extracted from dance videos are used for training as movement characteristics. During the model building phase, the model's generator module is used to achieve a basic mapping of music and dance movements and to generate gentle dance gestures. The identification module is used to achieve consistency between dance and music. The self-encoder module is used to make the audio function more representative. Experimental results on the DeepFashion dataset show that the generated model can synthesize the new view of the target person in any human posture of a given posture, complete the transformation of different postures of the same person, and retain the external features and clothing textures of the target person. Using a whole-to-detail generation strategy can improve the final video composition. For the problem of incoherent character movements in video synthesis, we propose to optimize the character movements by using a generative adversarial network, specifically by inserting generated motion compensation frames into the incoherent movement sequences to improve the smoothness of the synthesized video.

## 1. Introduction

The mapping of music to dance movements is a typical cross-modal generation task. Dance is an important part of the daily entertainment and life of people around the world, and it is closely related to music in its structure, artistic expression, and interpretation. In order to make dance and music fit better, choreographers need to create dance movements based on the characteristics of music [1–3]. Choreographers listen to the music, analyze the musical genre, characteristics, inner emotions or messages, and then design the corresponding dance movements based on the musical message [4]. This entire process is known as choreography, an art of collecting and organizing movement sequences based on music to reflect or express the dancer's thoughts and emotions. Researchers have used algorithms to simulate this process. In recent years, many applications related to music and dance have been introduced for educational and entertainment purposes, such as Jitterbug and MikuMikuDance. People can watch animated dance performances or even create their own [5–7].

A music-driven choreography algorithm would be useful in many areas, including assisting dancers in choreography, dance teaching and performance, animation, video games, robotics research, and more. However, few algorithms currently exist that can accurately match computer-generated dances to music [8]. Traditional dance generation algorithms typically construct a database of musical movements, which contain a large number of musical movement pairs. When a music clip is used as input, it is divided into several small music clips, each of which can be found in the database as the most similar clip. The system can then provide the corresponding dance movement candidates and combine them into a new dance movement. However, its limitation is that it cannot create new dance movements but can only arrange and combine them from its own existing dance movement database [9–11]. Dance data reflect the change of human body key point coordinates over time, which is typical of time series data, and thus has the characteristics of multi-scale, multi-dimensional, and dynamic correlation [12]. Dance video generation is one of the most interesting research directions in the field of video generation, which is a technique to study how to synthesize videos of target dance movements [13]. Dance video synthesis refers to giving a source video containing dance movements of a person, and transferring the dance movements in this video to the target person through deep learning techniques, so that the movements of the person in the final synthesized video are consistent with the postures of professional dancers in the source video, which is reflected in making amateur dancers have the level of professional dancers in the synthesized video [14–16].

The ability to transfer human movement poses between different dance videos and transfer graceful dance poses from original character to target character allows the audience to become dance masters and Internet celebrities in a short time. Related studies have shown that the use of deep neural network design and training techniques to transfer human movements from one video to another video character can produce personalized dance videos of subjects without dance experience. To address the above problems and characteristics of dance data, we created a custom music dance data set with about 270,000 frames of music and dance movements and extracted the key point coordinates of the iconic human skeleton as a feature of dance gestures using techniques for estimating human gestures. It proposes a music function encoder and a deep learning-based model for generating dance movements based on extracted dance functions, and music functions are trained end-to-end.

## 2. Methods

### 2.1. Human Posture Estimation

As shown in Figure 1, the cascaded pyramid network consists of two main parts, the first part of the network, named GlobalNet, which adopts the form of Feature Pyramid Network (FPN) to perform the initial detection of the human torso globally. GlobalNet effectively utilizes the different scales of feature maps output at different stages and can successfully locate the key points in the human torso, such as eyes, nose, and hands, which are easier to locate. The second part of the network, called RefineNet, is designed to build on the output of the first part of the network by fusing the features extracted from each layer of the GlobalNet network to perform a deeper and more refined detection. RefineNet is mainly used to detect keypoints that are influenced by external conditions or obscured, which can improve the final recognition of human keypoints. The model first extracts the 2D pose skeleton of the target person using a human pose detector (OpenPose), then learns the feature correspondence between images of two different domains, transforms the person image under the target pose, and optimizes the details of the generated image by adding a loss function for iterative training. Finally, we generate a high-quality image of the person with the target pose.

GlobalNet uses ResNet50 as the backbone of the network structure. The four solid rectangles on the left are Res2-Res5 in ResNet50, and the dashed rectangles on the right represent the feature fusion process through upsampling and summation [17]. GlobalNet has four layers, and each layer outputs one result, so the respective loss functions need to be calculated for each of the four different results. RefineNet takes the features extracted from GlobalNet at four different levels and inputs them into a number of residual blocks with different multiples of upsampling, and then the feature merge layer is used to stitch the feature maps of the same size from different layers. Then, the feature maps of the same size from different layers are stitched together in the feature merging layer to complete the feature fusion, and the final result is output by a residual block. The pose heat map is an important basis for detecting the target key points, and the convolutional neural network (CNN) is applied to pose detection to quantify the dependency of each key point of the human body and then obtain the heat map. The difficulty here is that since the two images are from different domains, their ImagePatch has a huge Domain Gap, and thus it is not possible to directly correspond the image blocks of the two types of images with some predefined distance metric (e.g., Euclidean distance).

In the first stage, the network outputs a set of confidence maps:

(1) $$\begin{array}{c} S=\sigma \left(F\right), \end{array}$$

and a set of partial affinity vector fields:

(2) $$\begin{array}{c} l\left(F\right)=\sigma \left(F\right)*T\left(f\right), \end{array}$$

where *F* and *L* are the expressions of the inferred results of the convolutional neural network at that stage based on the extracted feature maps, these two branches are trained iteratively separately, and each completed iteration can be considered as the completion of one stage. In the iterative process, the input of the branch network in the current stage is the feature map of the output of the previous stage network to the original image, and this feature repetition can produce more accurate predictions, as shown in the following Equation:

(3) $$\begin{array}{c} s\left(t\right)=\sigma *t\left(F,t,s\right),\;\forall \left.t\right.2,\\ l\left(t\right)=\sigma *t\left(F,t,l\right),\;\forall \left.t\right.2. \end{array}$$

In order to make the model converge iteratively during the training process and to improve the accuracy of the final prediction results for each branch, the respective loss functions are set at the end of each stage. The upper and lower branch networks have one loss function each, and the loss function is used to constrain the results between the true and predicted values. Among them, in order to solve some practical problems, such as some data sets are not fully labeled with all targets, the loss function is weighted spatially to strengthen the prediction results. The loss function of the up-and-down branching network in the first stage is:

(4) $$\begin{array}{c} f\left(t\right)=\sum_{i=1}^{q}t\left(F,t,l\right)\cdot \left\|s\left(t\right)-q\right\|,\\ f\left(l\right)=\sum_{i=1}^{q}t\left(F,t,l\right)\cdot \left\|l\left(t\right)-q\right\|. \end{array}$$

The model first encodes the connection between the joints of the human body through a feedforward network, which is then used to match the skeletal joints. After obtaining the key points of the human body in the image, the key points need to be correctly connected to construct the human skeleton map, specifically, the key points are clustered. A common clustering method is to connect the key points according to the distance between them. The key points of a single person can be connected according to the definition of the joint position of the human body, but for the case of multiple people in one image, it may be wrong to connect the key points of different people together when connecting the key points. To solve this problem, OpenPose proposes the part affinity vector field (PAF), which helps to connect the keypoints correctly by their distance and direction in prediction, and uses the Hungarian algorithm for clustering to get the optimal matching method of keypoints.

### 2.2. Human Pose Migration Based on Cross-Domain Correspondence

Human pose migration aims to convert the input conditional person image to a new image of that person in the target pose, and the appearance of the person and background texture of the generated image remain consistent with the source person image. Human pose migration has a wide range of applications in the fields of pedestrian re-identification, pose tracking, and behavior analysis. A difficult problem in existing methods for generating human images is that human images have more complex structures compared to other images, and therefore, the process of pose transformation often involves the deformation of larger nonrigid objects, such as joints and limbs. In addition, the appearance features and clothing textures of different characters are often different, leading to the fact that it is relatively easy to ignore these image feature detail information in the character images after pose migration. In this paper, we introduce a conditional generative adversarial network based on cross-domain correspondence learning. Firstly, the user clicks the pick file button, the system will start the file reading procedure and display the video file picking interface, waiting for the user to specify the video path.

The task of pose-guided human image generation can be understood as how to find the semantic correspondence between the pose labels and the person images [18]. It is shown that sparse sets of points corresponding between different images can be used for various image-processing tasks, such as TemplateMatching, Image Alignment, and Image Morphing, and this sparse cross-domain correspondence approach allows the input images of different domains or semantic classes to have relatively large differences in the sparse cross-domain correspondence for relatively large differences in the content and appearance of the input images of different domains or semantic categories. When finding a sparse set of cross-domain correspondences for different classes of images, it is often necessary to determine which points in one image are meaningful candidates for matching and to find their respective best counterparts in the other image, i.e., the goal of establishing cross-domain correspondences is to find matching pairs of points in the images, and these points should be located at important locations in two different images that contain key information. In general, finding the sparse correspondence between two images can be divided into two steps: extracting key points and performing matching. The key points of sparse matching form the basis of dense matching, and in the process of performing dense matching, this paper uses a pretrained convolutional neural network to extract and encode the deep feature maps, and then represents the feature mapping as a pyramid, specifically, the top layer of the feature pyramid is the last convolutional layer extracted features, and the bottom layer is the shallowest mapping.

### 2.3. Neural Network Model Building

The cross-domain correspondence network consists of two subnetworks, the first part is the Crossdomain Correspondence subnetwork, which is used to find the dense semantic correspondence between the pose skeleton and the person image [19]. The second part of the network is the Image RefinementNetwork, which attempts to generate the final image from the coarse image output of the previous network. Previous works usually choose pretrained deep learning models to match patch blocks in feature domains to find dense correspondences of images belonging to different domains. However, since the pretrained models are usually trained for a specific type of image dataset (e.g., ImageNet), the extracted features cannot be generalized to the semantic description of another image class to establish correspondence between different classes of images, such as image translation from semantically segmented images to real scenario images. To solve this problem, this paper adopts a cross-domain correspondence-based generative adversarial network, which maps the domains of the input images of different categories into a shared domain S, in which the features of two input images of different domains can be represented, and finds the semantic correspondence between the two different categories of images.

The domain alignment process is shown in Figure 2. Specifically, *x* and *y* are input to two feature pyramid networks, which use convolutional neural networks to extract multi-scale deep features of different classes of images, and then the extracted features are further sub-represented in the shared domain S as *x*, *y* ∈ *R* (H, W are feature space dimensions, C is the channel direction dimension) by the dense correspondence module. Then, the domain alignment can be expressed by the following equation:

(5) $$\begin{array}{c} x=ℑ\left\|l\left(t\right)-q\right\|,\\ y=ℑ\left\|x\left(t\right)-q\right\|. \end{array}$$

Specifically, the correlation matrix *M*, where each element is correlated in pairs of features, is calculated. The correlation matrix *M* is calculated as shown in the following equation:

(6) $$\begin{array}{c} M\left(x,y\right)=\frac{{\left[x\left(u\right)-y\left(u\right)\right]}^{T}\left[x\left(u\right)-y\left(u\right)\right]}{{\left[\left\|x\left(u\right)-y\left(u\right)\right\|\right]}^{T}\left\|x\left(u\right)-y\left(u\right)\right\|}. \end{array}$$

An effective way to do this is to train the cross-domain correspondence network together with the image enhancement network. During the training of the image enhancement network, the model is more likely to produce high-quality output if it refers to the correct correspondence regions in the training sample, which indicates that the network is able to learn accurate dense semantic correspondence in this way.

### 2.4. Data Input and Output Module Design

The data input and output module are mainly responsible for local video loading and online video entry, providing users with two ways to load test dance video data. So the data input and output module design will introduce two data input modes [20]. If the user clicks cancel or does not specify the correct video address or the video file is incorrectly read, the system will return the corresponding error message, as shown in Figure 3.

The skeleton detection module is internal to the system and is shielded from normal users. The system calls the skeleton detection module by default when performing character action training tasks or generation tasks. According to the video URL inputted by the data input process, the system will automatically read in the video file and use the ffmpeg tool to slice the video and scale it to the same size of 512*∗*1024; after getting the slice image collection, the system will automatically call the openpose detection function and send the slice image collection to the pose detection network to get the corresponding character skeleton and store the openpose output json file, which stores the key point information of the character. We redraw the character skeleton using our own drawing method, mainly using color to identify the front and back of the character, and weighted fusion of overlapping parts. The dance generation module mainly completes the task of generating the target character based on the user-specified dance source video. Firstly, the user needs to specify the target character, the system will have several target character action models, and the user can select the target character according to the drop-down list box; after selecting the specified character, the user also needs to specify the source video of the dance, that is, what kind of action he or she wants the target character to complete; the user clicks the open button; after selecting the appropriate video path, the system automatically reads in the video; then, the system automatically calls the skeleton detection module to parse the source video of the dance and present the skeleton map frame by frame; finally, the drawn skeleton map is input to the trained generator to get the corresponding action map of the target character. For the user to select the local video as the source video to generate the dance, the user needs to specify the URL address of the source video. When the user determines the source video file address, the system will get the absolute path of the file according to the source video selected by the user and pass the path to the data-processing module in order to execute the necessary processes for subsequent dance generation.

In order to improve the user control of the generative adversarial network and still improve the resolution and quality of the generated pictures of the generative adversarial network, we first use pairs of data for training, as shown in the previous section training with real sample pairs as (x, y) and false sample pairs as (G(x), y). This improvement then provides a correspondence between the appearance of the character and the skeleton for the generative network, and this has a wide range of applications; similar applications include hand sketching to generate pictures, coloring gray scale pictures, automatic coloring, etc. In pix2pixhd (which is also called pixel*∗*pixel HD), a coarse to fine generation network is used, but this application does not use that structure, but only borrows from the “coarse” network and uses its fine network. The generator network mainly generates 512*∗*1024 images and includes a series of self-encoding modules with residuals.

### 2.5. Discriminator Design

To be able to distinguish between high resolution real and synthetic images, the discriminator network needs a large field of view. A deeper network or a larger convolutional kernel can have a larger field of view, but this is also likely to lead to overfitting of the network and require more GPU memory for too many network parameters. In order to solve this problem, we use three discriminators, each with the same network structure but operating at different image scales {*d*1, *d*2, *d*3}, as proposed in the Pix2PixHD paper. Specifically, we downsample the real and synthetic high-resolution images by a factor of 2 and 4 to generate pyramidal image data at three scales. Discriminators *d*1, *d*2, *d*3 are trained to differentiate between real and synthetic images at three different scales. The discriminator has the same structure, but an operation at the coarsest scale has the largest field of perception. It has more of a global view of the image and guides the generator to generate a globally continuous image. On the other hand, the discriminator at the smallest scale encourages the generator to generate finer details. This also makes it easier to train coarse-to-fine generators. To extend the low resolution model to meet the higher resolution, it only needs to add a discriminator in the most fine-grained layer, rather than retraining from the skeleton. The input to each discriminator network is an image at a different scale, and the results are finally fed into a patch-based generative adversarial loss. This achieves a discriminator network with a large perceptual field. The original generative adversarial network evolves into a multi-task generative adversarial network (see loss function design). The multi-scale discriminator differs only in the size of the input images; otherwise, all structures are the same. In order to solve the quality and resolution problems of the generated image, we used the pix2pixhd structure to generate a high resolution image.

## 3. Dance Tracking Algorithm Implementation

### 3.1. Discriminator Loss

Firstly, the loss function in the danceTrans algorithm is mainly divided into generator loss and discriminator loss, and the generator loss mainly includes adversarial loss, VGG-based perceptual loss, and feature matching loss. Adversarial loss has become a popular choice for many image-to-image tasks, because the discriminator can learn a trainable loss function and automatically adapt to the differences between the generated and real images in the target domain. The feature matching loss is more important to ensure that the generated model does not oscillate too much. Moreover, it has been shown experimentally that increasing the vgg perceptual loss can slightly improve the generation results in some cases. The discriminator loss mainly includes the loss of real image pairs and the loss of false image pairs, i.e., the loss caused by discriminating real images into false ones and discriminating false images into real ones. As shown in Figure 4, the loss values saved during the training process are visualized, and the content of this figure is the image visualized after all generator losses are superimposed, and it can be seen that the generator losses will have large jitter during the training of the generative adversarial network, and this problem will be significantly alleviated after multiple rounds of training. However, during the training process, there is often a sudden jump in the value of a loss. We specifically analyze the problem here, mainly in the synthesis of the back image of the character, and the front image of the distribution gap is large, so the synthesis does not distinguish between the front and back of the character, resulting in the loss value jitter. Experimental results on the DeepFashion dataset show that the generative model is able to synthesize a new view of the target person in an arbitrary human pose given the pose, complete different pose transformations of the same person, and preserve the external features and clothing textures of the target person. Using a whole-to-detail generation strategy can improve the final video composition.

### 3.2. System Effect Comparison

The dance generation algorithm danceTrans proposed only in this system is based on the Pix2PixHD algorithm, while this subsection makes a systematic comparison between the two algorithms, mainly introducing two image quality assessment metrics as well as comparing the two models to generate image quality for the same skeleton. The goal of the generative model is to give the model the ability to generate data and to match the observed data. Therefore, the distance between the observed probability pw of the actual sampled data and the probability *p* of the data distribution of the generated model can be used as an evaluation metric for the performance of the generated model. However, it is very difficult to define a suitable evaluation metric for the generative model, and it is known that it can be measured using the likelihood or estimated by sampling the sample importance. However, the likelihood is not a good measure of the difference between the two distributions because it relies heavily on the assumption of noise in the actual true sample data and is ruled by a single sample. FID is sensitive to pattern collapse. As shown below, the distance increases with the simulated missing pattern. This is shown in Figure 5. One of the most significant improvements is the pyramidal approach, where a low-resolution image is output first, and then the previously output low-resolution image is used as input to another generation network to continue generating a better-detailed, higher-resolution image.

FID is more robust than ssim evaluation. If the model generates only one image per class, the calculated distances will be large. Therefore, FID gives a better measure of image diversity. FID has some fairly high bias in some cases, but the variance is small. By calculating the FID between the training and test datasets, we should expect the FID to be zero, since both are real images. In the system structure design section, we design the structure of the whole system into three layers: application layer, logic layer, and data layer, and design the functional flow of each module and the data structure design of the whole system in detail. We designed and implemented a dance generation algorithm based on deep convolutional generative adversarial network. We elaborated a flowchart that can manipulate the source character to perform a series of standard movements based on a target video of a given professional dancer to synthesize a new dance video. We use generative adversarial network techniques and image generation techniques to transfer the professional dance performance to the target character. The algorithm uses the human skeleton map as an intermediate representation between the source and target videos.

### 3.3. Dance Tracking Authenticity

First, we investigated whether the dances generated by the models were realistic and credible. The score of each model is calculated based on the average of the scores of the scorers for the 15 videos, and then the scores of all the scorers are averaged to obtain the realism score of each model, as shown in Figure 6. In the requirement analysis of the system, this paper provides a detailed description of the requirements of the dance generation system, pointing out the application scenario of this system as well as describing the use cases of this system and the functions belonging to it.

We set model one to be the LSTM-PCA model, model two to be the LSTM-PCA + Discriminator model, model three to be the Generator part of our dance generation model, model four to be the Generator + Discriminator model, and model five to be the Generator + Discriminator + Autoencoder model. Autoencoder model. As can be seen from the table, our Generator series models are better than the other models in terms of realism. Specifically, Model 1 scored 3.61, Model 2 scored 5.43, Model 3 scored 6.90, Model 4 scored 7.85, and Model 5 scored 8.52. The dances generated by the models were then scored by the users for their consistency with the music. Since the dataset contains three types of dances, Kpop, Poppin, and Hiphop, each user is asked to score each of the three types of dances generated by each model on the basis of whether the dances generated by the models match the music or not. Finally, the average of the music consistency scores for each type of dance was calculated based on the scores of all users.

## 4. Discussion

### 4.1. Posture Consistency

As can be seen from Figure 7, in terms of musical consistency, our Generator series model is better than the other models. In terms of data, the musical consistency of the Kpop dataset is higher than that of the other categories of dances, which may be due to the fact that the data within the datasets of the other two dances are more varied, model 2 scored 5.61 on the Kpop dataset, 4.32 on the Poppin dataset, and 4.21 on the Hiphop dataset; model 3 scored 6.54 in Kpop dataset, 5.32 in Popin dataset, and 5.39 in Hiphop dataset.

Model 4 scored 8.01 in the Kpop dataset, 7.21 in the Poppin dataset, and 7.45 in the Hiphop dataset; Model 5 scored 9.01 in the Kpop dataset, 7.98 in the Poppin dataset, and 7.32 in the Hiphop dataset. In summary, our model achieves the best user ratings in terms of dance authenticity and music consistency relative to other models.

### 4.2. Image Quality Assessment Results

As shown in Figure 8, the scores are better even for single frame results using the global content discriminator and the local time discriminator. The addition of the pose perception deficit makes the pose plausible and then the transfer of the different pose to the frame may lead to a decrease in the score. In addition, more significant differences can be observed in our videos. This reflects the soundness and effectiveness of the design of our scheme in the feature extraction phase and the design in the model building phase.

The experimental results on the loss function values of the dance generation model show that in the feature extraction stage, removing the wrong dance gesture frames can effectively reduce the loss and improve the prediction ability of the model, and interpolating the missing values is also beneficial to the final dance gesture generation. In the model building stage, our Generator + Discriminator + Autoencoder-based model has higher loss values than the pure Generator model, but it can generate dances that fit the music better, reflecting the multimodality of the Generator and Discriminator combination; when comparing with other baselines, our model has lower loss values than the pure LSTM series model and generates better results. The experimental results on the evaluation of dance gesture sequences for the dance generation model show that our model generates dance gestures that are closest to the real dance gestures compared to other models, both for the music in the training set and the music in the test set. This also reflects that our model has the best sequence generation compared to other models. The synthesized live-action effect is also the best, as shown in Figure 9.

In the model building phase, the effect of different modules on the model loss is analyzed under the premise of using filtered out erroneous data, using cadence features and interpolation of missing values. The generator based on the tacotron2 model has a better fit for the sequences and the losses are relatively low, probably thanks to the fact that the generator decoder is an autoregressive model. In the case of adding Discriminator, the loss value is slightly larger than the case without Discriminator. This is to be expected because adversarial training causes the generator to generate a new sequence that does not necessarily match the original dance gesture sequence, and this new sequence may deviate more from the Groundtruth than the dance gesture predicted by optimizing only the Euclidean loss. A comparative analysis of the three types of models mentioned above shows that the Autoencoder module has a significant effect on the loss of the model.

## 5. Conclusion

Computer vision technology has been more and more widely used in human life, bringing great changes to people's lifestyles. This paper focuses on image and video synthesis based on human pose key points. In this paper, we focus on the image and video synthesis based on the key points of human pose, and decompose the pose transformation of a person into two subtasks, i.e., feature extraction of joint points using human pose estimation method and image synthesis using generative adversarial network. Finally, the proposed method is experimented on the dataset and the results are analyzed and discussed. The main contributions of the paper can be summarized as follows: to address the problems of the YouTube Dancer-18 dataset, such as fewer training samples, insufficient data diversity, and low video resolution, the paper supplements more single dance videos with higher definition and more dance types, and the new dataset is well able to train various deep learning models for human motion transfer tasks. Experimental results on the DeepFashion dataset show that the generative model is able to synthesize a new view of the target person in an arbitrary human pose given the pose, complete different pose transformations of the same person, and preserve the external features and clothing textures of the target person. Using a whole-to-detail generation strategy can improve the final video composition. For the problem of incoherent character movements in video synthesis, we propose to optimize the character movements by using a generative adversarial network, specifically by inserting generated motion compensation frames into the incoherent movement sequences to improve the smoothness of the synthesized video.

## Figures and Tables

**Figure 1:** Pose estimation model.

**Figure 2:** Cross-domain correspondence network framework diagram.

**Figure 3:** Flowchart of the Get Local Video module.

**Figure 4:** Generator loss curve.

**Figure 5:** Relationship between FID metric values and image quality.

**Figure 6:** Dance authenticity scoring chart.

**Figure 7:** Music consistency scoring chart.

**Figure 8:** Image quality assessment score.

**Figure 9:** Training frames during the bin center.

## Data Availability

The data used to support the findings of this study are included within the article.
